The article "Long noncoding RNA NR2F1-AS1 promotes the malignancy of non-small cell lung cancer via sponging microRNA-493-5p and thereby increasing ITGB1 expression" was retracted in 2024. Reasons: plagiarized images; overlap with other authors' work; signs of a paper mill.

# Long noncoding RNA NR2F1-AS1 promotes the malignancy of non-small cell lung cancer via sponging microRNA-493-5p and thereby increasing ITGB1 expression

**DOI:** 10.18632/aging.103564

**Published:** 2020-08-07

**Authors:** Chan Zhang, Shangjie Wu, Rong Song, Changming Liu

**Affiliations:** 1 Department of Respiratory Medicine, The Second Xiangya Hospital of Central South University, Changsha 410000, Hunan, China; 2 Department of Respiratory Medicine, The Fourth Hospital of Changsha, Changsha 410006, Hunan, China; 3 Department of Anesthesiology, The Second Xiangya Hospital of Central South University, Changsha 410000, Hunan, China; 4 Department of Infectious Diseases, The First Hospital of Changsha, Changsha 410000, Hunan, China

**Keywords:** NR2F1 antisense RNA 1, microRNA-493-5p, ceRNA, non-small cell lung cancer

## Abstract

Several studies have reported that the long noncoding ribonucleic acid (lncRNA) NR2F1 antisense RNA 1 (NR2F1-AS1) affects multiple cellular pathways that are involved in tumorigenesis and tumor progression. The present study aimed to detect NR2F1-AS1 expression in non-small cell lung cancer (NSCLC), investigate the role of NR2F1-AS1 in promoting the tumorigenic behavior of NSCLC cells, and elucidate the mechanism underlying the effect of NR2F1-AS1 on NSCLC progression. Our results showed that NR2F1-AS1 expression was upregulated in NSCLC cells, and notably, its upregulation was correlated with adverse clinical characteristics and shorter overall survival in patients with NSCLC. The absence of NR2F1-AS1 functionally decreased NSCLC cell proliferation, migration, and invasion and promoted tumor cell apoptosis. In addition, the tumor growth of NSCLC cells *in vivo* was inhibited after NR2F1-AS1 silencing. Mechanistically, NR2F1-AS1 functioned as a competing endogenous RNA for miR-493-5p and consequently increased ITGB1 expression. Rescue assays further validated that an increased output of the miR-493-5p/ITGB1 axis could neutralize the regulatory impact of NR2F1-AS1 knockdown on the malignant phenotype of NSCLC cells. In summary, the NR2F1-AS1/miR-493-5p/ITGB1 pathway initiates pro-oncogenic behavior in NSCLC tumor progression, and the NR2F1-AS1/miR-493-5p/ITGB1 axis may provide new molecular targets for anticancer therapy against NSCLC.

## INTRODUCTION

Lung cancer has become the most prevalent leading cause of cancer-related mortality worldwide [1]. Annually, approximately 2.1 million new cases of lung cancer are diagnosed and 1.8 million deaths are caused by this disease worldwide [1]. Non-small cell lung cancer (NSCLC) is the most frequent histological subtype of lung cancer, accounting for approximately 85% of all lung cancer cases [2]. The 5-year relative survival rate of patients with NSCLC is approximately 15%, which has remained unchanged over the past few decades, despite the substantial advancements in diagnostic techniques and therapies [3]. Moreover, difficulty in the diagnosis of NSCLC at the early stage remains another challenge; most patients with NSCLC are diagnosed at middle and advanced stages [4]. Multiple factors play a role in the occurrence and development of NSCLC, including oncogenic gene activation, tumor-suppressing gene inactivation, tobacco smoking, heterogeneity, and radon gas and asbestos exposure [5–7]. Despite the prevalence of NSCLC and the associated high mortality rate, the detailed molecular events associated with its tumorigenic behaviors have not yet been well elucidated. Therefore, it is imperative to further investigate the etiology of this disease and to determine the accurate pathogenetic mechanisms associated with it, which may aid in the development of unique diagnostic biomarkers and therapeutic targets.

Long noncoding ribonucleic acids (lncRNAs) comprise a family of transcripts of >200 nucleotides that have no protein-coding ability [8]. Currently, >3,000 lncRNAs have been verified in the human genome [9]. In recent years, lncRNAs have been validated as novel gene regulators and they exert their effects on gene expression via different mechanisms, including chromosome remodeling and transcriptional and post-transcriptional processing [10]. Numerous recent discoveries have demonstrated the indispensable roles of lncRNAs in microorganisms, plants, animals, and humans [11]. LncRNAs have gained wide attention owing to their role in tumor initiation and progression [12–14]. Differentially expressed lncRNAs have been reported in various human cancer types, including NSCLC [15–17]. The normal function of a considerable amount of lncRNAs is dysregulated in NSCLC, thus demonstrating their critical roles in regulating malignant physiological or pathological cellular processes via pro- or anti-oncogenic actions [18–20]. Several studies have demonstrated their potential application in the diagnosis, prognosis, and therapy of NSCLC [21–23]. Despite the wide-ranging functions of lncRNAs, a detailed examination regarding the functions and relevant mechanism of cancer-related lncRNAs in NSCLC has not been extensively studied and thus warrants an in-depth investigation.

Although several studies have reported that the lncRNA termed NR2F1 antisense RNA 1 (NR2F1-AS1) affects various cellular processes that initiate tumorigenesis and promote tumor progression [24–29], studies reporting the expression and role of NR2F1-AS1 in NSCLC and the mechanisms underlying its pro-oncogenic activities in NSCLC progression are limited. Therefore, the present study aimed to determine NR2F1-AS1 expression in NSCLC cells, investigate the roles of NR2F1-AS1 in NSCLC cells, and elucidate the mechanisms underlying the effect of NR2F-AS1 on NSCLC progression. To the best of our knowledge, this is the first study to focus on NR2F1-AS1 expression in NSCLC cells, and we believe that the findings may offer valuable clues for diagnosis and therapy of NSCLC.

## RESULTS

### High NR2F1-AS1 expression is associated with poor clinical outcomes in NSCLC

To examine whether NR2F1-AS1 plays a role in NSCLC, quantitative reverse transcription–PCR (RT–qPCR) was initially employed to determine NR2F1-AS1 expression in 73 pairs of NSCLC tissues and matched adjacent normal tissues. The data showed that NR2F1-AS1 expression was evidently upregulated in NSCLC tissues compared with that in matched adjacent normal tissues (Figure 1A). Consistent with the finding from tissue samples, a substantial increase in NR2F1-AS1 expression was confirmed in all the five NSCLC cell lines compared with that in the normal nontumorigenic bronchial epithelium cell line BEAS-2B (Figure 1B).

**Figure 1:** **NR2F1-AS1 is highly expressed in NSCLC and is linked with poor NSCLC clinical outcomes.** (**A**) Relative NR2F1-AS1 expression in 73 pairs of NSCLC tissues and matched adjacent normal tissues was evaluated by RT–qPCR. (**B**) RT–qPCR analysis was employed to assess the expression patterns of NR2F1-AS1 in five NSCLC cell lines and in the normal nontumorigenic bronchial epithelium cell line BEAS-2B. (**C**) Kaplan–Meier survival curves correlated with the expression level of NR2F1-AS1. High NR2F-AS1 expression relates to shorter overall survival rate NSCLC patients (P = 0.024). *P < 0.05 and **P < 0.01.

The median NR2F1-AS1 expression in NSCLC tissues was defined as the cut-off value, and all the 73 patients with NSCLC were accordingly classified into either low NR2F1-AS1 (n = 36) or high NR2F1-AS1 (n = 37) expression groups. Investigation of the clinical characteristics of the 73 patients with NSCLC revealed that an elevated NR2F1-AS1 expression was evidently associated with tumor size (P = 0.005), tumor–node–metastasis (TNM) stage (P = 0.038), and lymph node metastasis (P = 0.025), which are indicative of poor prognostic outcomes (Table 1). In addition, the overall survival of patients with high NR2F1-AS1 expression was shorter than that of patients with low NR2F1-AS1 expression (Figure 1C, P = 0.024). Taken together, these data characterized the abnormal NR2F1-AS1 overexpression in tissue samples from patients with NSCLC and suggested an evident association between NR2F1-AS1 expression and NSCLC progression.

**Table 1:** Correlations between NR2F1-AS1 and clinical characteristics of 73 NSCLC patients.

**Characteristics**	**NR2F1-AS1 Level**		**P**
	**High (n = 37)**	**Low (n = 36)**	
**Gender**			0.334
Male	26	21	
Female	11	15	
**Age (years)**			0.346
< 60	13	17	
≥ 60	24	19	
**Smoking history**			0.634
Yes	16	13	
No	21	23	
**Tumor size (cm)**			0.005
< 3	20	31	
≥ 3	17	5	
**Differentiation**			0.778
High and Moderate	7	8	
Poor	30	28	
**TNM stage**			0.038
I+II	22	30	
III+IV	15	6	
**Lymph node metastasis**			0.025
Negative	24	32	
Positive	13	4	

Abbreviations: TNM, tumor–node–metastasis;

### Knockdown of NR2F1-AS1 decreased the tumorigenic behavior of NSCLC cells

H460 and A549 cell lines demonstrated higher NR2F1-AS1 expression than the other three NSCLC cell lines; therefore, we selected these two cell lines for subsequent experiments. To investigate whether NR2F1-AS1 expression influences the tumorigenic behavior of NSCLC cells, three different small interfering RNAs (siRNAs) designed to silence NR2F1-AS1 were transfected into H460 and A549 cell lines and RT–qPCR was performed to evaluate the silencing efficiency. The results showed that transfection with all the three siRNAs resulted in efficient NR2F1-AS1 knockdown (Figure 2A). si-NR2F1-AS1#1, which possessed the highest transfection efficiency, was used in functional assays (henceforth, termed as si-NR2F1-AS1).

**Figure 2:** **Reduction in NR2F1-AS1 expression results in attenuated proliferation, migration, and invasion as well as promoted apoptosis of H460 and A549 cells.** (**A**) H460 and A549 cells were transfected with three different siRNAs targeting NR2F1-AS1 and si-NC, and the level of NR2F1-AS1 was determined by RT–qPCR. (**B**) CCK-8 assay demonstrated that silencing of NR2F1-AS1 suppressed the proliferative potential of H460 and A549 cells. (**C**) Flow cytometry analysis showed that the apoptosis in H460 and A549 cells was promoted after si-NR2F1-AS1 transfection. (**D**, **E**) Cell migration and invasion assays revealed that the migratory and invasive capacities of H460 and A549 cells were hindered by NR2F1-AS1 inhibition (x200 magnification). *P < 0.05 and **P < 0.01.

Cell counting kit (CCK)-8 assay was conducted to assess the proliferation rates of H460 and A549 cells following NR2F1-AS1 silencing. Transfection with si-NR2F1-AS1 notably inhibited the proliferative potential of H460 and A549 cells (Figure 2B). In addition, NR2F1-AS1 knockdown increased the apoptotic H460 and A549 cell population, as shown in Figure 2C. Furthermore, the migration (Figure 2D) and invasion (Figure 2E) potentials of H460 and A549 cells transfected with si-NR2F1-AS1 were considerably decreased compared with those of cells transfected with si-NC, as evidenced by cell migration and invasion assays. Overall, these results indicated that NR2F1-AS1 plays an important role in the oncogenicity of NSCLC.

### NR2F1-AS1 operates as a molecular sponge of miR-493-5p in NSCLC cells

To illuminate the mechanisms underlying the tumor-promoting roles of NR2F1-AS1, its localization in NSCLC cells was examined via subcellular fractionation. NR2F1-AS1 was mostly located in the cytoplasm of H460 and A549 cells (Figure 3A), suggesting that this lncRNA exerts its regulatory actions posttranscriptionally. The most acknowledged mechanism of cytoplasmic lncRNAs is that they are implicated in the regulation of gene expression by acting as competitive endogenous RNAs (ceRNAs) for miRNAs [30–32]. To determine whether NF2F1-AS1 functions as a ceRNA, we performed bioinformatics analysis to search for putative miRNAs for NR2F1-AS1 and found that miR-493-5p comprised potential complementary binding sequences for NR2F1-AS1 (Figure 3B). Considering its aberrant downregulation in NSCLC and anti-oncogenic actions during NSCLC progression [33], miR-493-5p was selected for additional experimental verification.

**Figure 3:** **NR2F1-AS1 directly interacts with miR-493-5p in NSCLC cells as a ceRNA.** (**A**) The subcellular distribution of NR2F1-AS1 in the cytoplasm or nucleus of H460 and A549 cells. (**B**) The wild-type binding site of miR-493-5p in NR2F1-AS1 was predicted by StarBase 3.0. The mutant binding sequences were also shown. (**C**) The efficiency of miR-493-5p mimic transfection in H460 and A549 cells was examined by RT–qPCR. MiR-NC served as the control. (**D**) The wt-NR2F1-AS1 or mut-NR2F1-AS1 reporter plasmids alongside miR-493-5p mimic or miR-NC were cotransfected into H460 and A549 cells. Luciferase reporter assay indicated that miR-493-5p could directly bind to NR2F1-AS1 in H460 and A549 cells. (**E**) RIP assay revealed the enrichment of NR2F1-AS1 and miR-493-5p in RNA immunoprecipitation with AGO2 antibody. (**F**) MiR-493-5p expression in 73 pairs of NSCLC tissues and matched adjacent normal tissues was determined via RT–qPCR. (**G**) Pearson's correlation coefficient was utilized to test the relationship between NR2F1-AS1 and miR-493-5p in the 73 NSCLC tissues (r = −0.6435, P < 0.0001). (**H**) MiR-493-5p expression was analyzed by RT–qPCR in H460 and A549 cells after transfection with si-NR2F1-AS1 or si-NC. *P < 0.05 and **P < 0.01.

To confirm the above hypothesis, luciferase and RNA immunoprecipitation (RIP) assays were performed to determine the actual interaction between NR2F1-AS1 and miR-493-5p in NSCLC cells. First, H460 and A549 cells were transfected with miR-493-5p mimic and RT–qPCR confirmed the upregulation of miR-493-5p expression (Figure 3C). As revealed by the luciferase reporter assay, exogenous miR-493-5p expression resulted in a noticeable decrease in the luciferase activity of wt-NR2F1-AS1 reporter plasmid carrying the wild-type miR-493-5p binding site; however, the luciferase activity of mut-NR2F1-AS1 remained unaltered in response to miR-493-5p overexpression (Figure 3D). Notably, the results of RIP assay showed that miR-493-5p and NR2F1-AS1 were greatly enriched in the anti-argonaute 2 (AGO2) group compared with that observed in the IgG control group (Figure 3E).

To further evaluate the association between NR2F1-AS1 and miR-493-5p, RT–qPCR was performed to measure miR-493-5p expression in tumor tissues and matched adjacent normal tissues collected from 73 patients with NSCLC. The miR-493-5p expression in NSCLC tumor tissues was lower than that in adjacent normal tissues (Figure 3F). Furthermore, Pearson's correlation coefficient revealed that NR2F1-AS1 expression was inversely correlated with miR-493-5p expression in the 73 NSCLC tissues (Figure 3G; r = −0.6435, P < 0.0001). Conversely, when si-NR2F1-AS1 was transfected into H460 and A549 cells, miR-493-5p expression was considerably increased upon NR2F1-AS1 downregulation compared with that observed in cells transfected with si-NC (Figure 3H). Taken together, these results suggested that NR2F1-AS1 functions as a molecular sponge for miR-493-5p in NSCLC cells.

### NR2F1-AS1 positively regulates the ITGB1 expression in NSCLC cells by sponging miR-493-5p

Because ITGB1 is the direct target of miR-493-5p in NSCLC cells, we determined whether NR2F1-AS1 competitively binds to miR-493-5p and consequently decreases miR-493-5p-mediated ITGB1 deregulation and/or translation suppression. Interference of NR2F1-AS1 expression led to an apparent downregulation of ITGB1 mRNA (Figure 4A) and protein (Figure 4B) expression in H460 and A549 cells. In addition, RT–qPCR revealed that the mRNA level of ITGB1 was increased in NSCLC tissues compared with that in the adjacent normal tissues (Figure 4C). Furthermore, a clear positive association was observed between NR2F1-AS1 and ITGB1 mRNA levels in the 73 NSCLC tissues (Figure 4D; r = 0.5704, P < 0.0001), as shown by Pearson's correlation coefficient. Rescue assays were further applied to examine whether NR2F1-AS1 positively regulates ITGB1 expression in a manner that was inversely dependent on miR-493-5p expression. MiR-493-5p inhibitor or NC inhibitor along with si-NR2F1-AS1 was cotransfected into H460 and A549 cells. First, the efficiency of miR-493-5p inhibitor was determined using RT–qPCR (Figure 4E). Following cotransfection, RT–qPCR and western blotting were performed, and the results revealed that the knockdown of NR2F1-AS1 caused a substantial decrease in ITGB1 mRNA (Figure 4F) and protein (Figure 4G) levels. Conversely, ITGB1 expression was recovered in NR2F1-AS1-deficient H460 and A549 cells following miR-493-5p inhibitor cotransfection. Taken together, these results indicated that NR2F1-AS1 acts as a ceRNA for miR-493-5p to positively regulate ITGB1 expression in NSCLC cells.

**Figure 4:** **NR2F1-AS1-mediated sponging of miR-493-5p increases ITGB1 expression in H460 and A549 cells.** (**A**, **B**) The mRNA and protein levels of ITGB1 in H460 and A549 cells transfected with si-NR2F1-AS1 or si-NC were measured by RT–qPCR and western blotting, respectively. (**C**) ITGB1 mRNA expression in 73 pairs of NSCLC tissues and matched adjacent normal tissues was determined by RT–qPCR. (**D**) Expression correlation between NR2F1-AS1 and ITGB1 mRNA in the 73 NSCLC tissues was identified by Pearson's correlation coefficient (r = 0.5704, P < 0.0001). (**E**) MiR-493-5p inhibitor or NC inhibitor was transfected into H460 and A549 cells, and the efficiency of miR-493-5p silencing was verified by RT–qPCR. (**F**, **G**) MiR-493-5p inhibitor or NC inhibitor was cotransfected into H460 and A549 cells with si-NR2F1-AS1. Expression change in ITGB1 mRNA and protein levels was evaluated by RT–qPCR and western blotting, respectively. *P < 0.05 and **P < 0.01.

### Increasing miR-493-5p/ITGB1 output eliminates the influences of NR2F1-AS1 knockdown on the aggressive phenotypes of NSCLC cells

To explore the roles of the miR-493-5p/ITGB1 axis in NR2F1-AS1-mediated aggressive phenotypes of NSCLC cells, si-NR2F1-AS1-treated H460 and A549 cells were further transfected with an miR-493-5p inhibitor or NC inhibitor. CCK-8 assay and flow cytometry analysis indicated that the inhibition of miR-493-5p reversed the impacts of NR2F1-AS1 knockdown on the proliferation (Figure 5A) and apoptosis (Figure 5B) of H460 and A549 cells. Additionally, cell migration and invasion assays illustrated that the depletion of NR2F1-AS1 suppressed the migratory (Figure 5C) and invasive (Figure 5D) abilities of H460 and A549 cells and that this suppression was recovered after miR-493-5p inhibition. Furthermore, rescue assays were conducted to verify the functional relevance between NR2F1-AS1 and ITGB1 in NSCLC cells. Furthermore, transfection with recombinant pcDNA3.1 ITGB1 overexpression plasmid pc-ITGB1 greatly increased the ITGB1 protein levels in H460 and A549 cells (Figure 6A), following which pc-ITGB1 or pcDNA3.1 plasmid along with si-NR2F1-AS1 was cotransfected into H460 and A549 cells. The decrease in cell proliferation (Figure 6B) and increase in cellular apoptosis (Figure 6C) as a result of NR2F1-AS1 silencing was restored using pc-ITGB1 treatment in H460 and A549 cells. Furthermore, the migration (Figure 6D) and invasion (Figure 6E) of H460 and A549 were inhibited by NR2F1-AS1 downregulation, and this effect was eliminated after cotransfection with pc-ITGB1. These data suggested that NR2F1-AS1 regulates the tumorigenic behavior of NSCLC cells and that this activity is dependent on the miR-493-5p/ITGB1 axis.

**Figure 5:** **Repression of miR-493-5p reverses the impacts of NR2F1-AS1 silencing on NSCLC cells.** H460 and A549 cells were transfected with si-NR2F1-AS1 in combination with miR-493-5p inhibitor or NC inhibitor. (**A**, **B**) Rescue effects of miR-493-5p inhibition on si-NR2F1-AS1-mediated inhibition of cell growth and promotion of apoptosis in H460 and A549 cells were explored by CCK-8 assay and flow cytometry analysis. (**C**, **D**) Rescue effects of miR-493-5p inhibition on si-NR2F1-AS1-mediated suppression of cell migration and invasion in H460 and A549 cells were evaluated by cell migration and invasion assays (x200 magnification). *P < 0.05 and **P < 0.01.

**Figure 6:** **Reintroduction of ITGB1 eliminates the functions of NR2F1-AS1 knockdown on NSCLC cells.** (**A**) Western blotting illustrated the protein level of ITGB1 in pc-ITGB1 or pcDNA3.1-transfected H460 and A549 cells. (**B**, **C**) CCK-8 assay and flow cytometry analysis showed the proliferation and apoptosis of H460 and A549 cells after cotransfection with si-NR2F1-AS1 and pc-ITGB1 or pcDNA3.1. (**D**, **E**) Cell migration and invasion assays detected the migratory and invasive abilities of H460 and A549 cells treated as described above (x200 magnification). *P < 0.05 and **P < 0.01.

### NR2F1-AS1 knockdown restrains NSCLC tumor growth *in vivo*

To determine the impact of NR2F1-AS1 on NSCLC tumor growth *in vivo*, xenograft tumor assays were performed by subcutaneously inoculating H460 cells with stable transfections of sh-NR2F1-AS1 or sh-NC into nude mice. The volume of tumor xenografts was monitored every week. The growth of tumor xenografts in the sh-NR2F1-AS1 group was noticeably suppressed compared with that observed in the sh-NC group (Figure 7A, 7B). Consistent with the visible growth stated above, the weight of tumor xenografts in sh-NR2F1-AS1-transfected nude mice was lower than that of xenografts in sh-NC-transfected mice (Figure 7C). The mice were sacrificed after 5 weeks, and total RNA and protein were isolated and subjected to analysis of NR2F1-AS1, miR-493-5p, and ITGB1 expression. RT–qPCR confirmed that NR2F1-AS1 expression was strikingly suppressed (Figure 7D) and miR-493-5p expression was promoted (Figure 7E) in the tumor xenografts derived from sh-NR2F1-AS1-transfected H460 cells. Furthermore, the ITGB1 protein level was decreased in the tumor xenografts injected with sh-NR2F1-AS1 (Figure 7F). These results suggested that NR2F1-AS1 knockdown restrains tumor growth of NSCLC cells via the miR-493-5p/ITGB1 axis.

**Figure 7:** **NR2F1-AS1 silencing impairs NSCLC tumor growth *in vivo*.** (**A**) Growth curves of volumes in tumor xenografts were determined based on tumor volume measured every week for 5 weeks. (**B**) Tumor xenografts derived from sh-NR2F1-AS1 or sh-NC stably transfected H460 cells were collected and photographed. (**C**) The weights of tumor xenografts in sh-NR2F1-AS1 and sh-NC groups were measured at 5 weeks after cell tumor cell inoculation. (**D**, **E**) RT–qPCR was utilized to detect expression levels of NR2F1-AS1 and miR-493-5p in tumor xenografts derived from sh-NR2F1-AS1 or sh-NC stably transfected H460 cells. (**F**) Western blotting was employed to determine ITGB1 protein expression in tumor xenografts obtained from sh-NR2F1-AS1 and sh-NC groups. **P < 0.01.

## DISCUSSION

The complexity of NSCLC severely limits the research regarding its pathogenesis and the development of novel therapies [34, 35]. Recently, an increasing number of studies have reported the aberrations of lncRNAs in NSCLC and have stated that these aberrations are essential for tumor incidence and development [36–38]. In view of the above, identification of cancer-associated lncRNAs and determination of their functional roles in NSCLC pathogenesis may aid in the development of new targets for potential therapeutic agents. Despite the numerous lncRNAs identified in the human genome, their detailed roles in NSCLC progression and relevant mechanisms of action require further research [9]. In the present study, we determined the expression profile of NR2F1-AS1 in NSCLC and evaluated its clinical significance for patients with NSCLC. The regulatory impact of NR2F1-AS1 on the tumorigenic behavior of NSCLC cells was investigated *in vitro* and *in vivo*. Furthermore, the molecular events via which NR2F1-AS1 regulates NSCLC cell oncogenicity were elucidated in detail.

NR2F1-AS1 expression is reported to be upregulated in osteosarcoma and this upregulation is closely correlated with advanced clinical stage and distant metastasis [24]. Patients with osteosarcoma exhibiting high NR2F1-AS1 expression had shorter overall survival rates than those exhibiting low NR2F1-AS1 expression [24]. Furthermore, high NR2F1-AS1 expression has been reported in esophageal squamous cell carcinoma [25], hepatocellular carcinoma [26], endometrial cancer [27], and papillary thyroid carcinoma [28, 29]. However, only few studies to date have focused on the enrichment and function of NR2F1-AS1 in NSCLC. Here we determined the expression profile of NR2F1-AS1 in NSCLC tissues and cell lines, revealing the aberrant upregulation of NR2F1-AS1 expression in NSCLC. Importantly, elevated NR2F1-AS1 expression was found to be associated with adverse clinical characteristics and poor clinical outcomes in patients with NSCLC.

NR2F1-AS1 plays a significant role in tumor biology. For instance, a reduction in NR2F1-AS1 expression leads to decreased osteosarcoma cell proliferation, migration, and invasion *in vitro* and decreased tumor growth *in vivo* [24]. Additionally, the interference of NR2F1-AS1 expression reportedly increases cell apoptosis and induces cell cycle arrest in osteosarcoma [24]. Further, NR2F1-AS1 exerts tumor-promoting roles in esophageal squamous cell carcinoma progression and is implicated in the regulation of cellular viability, colony formation, proliferation, migration, invasion, and sphere-forming ability [25]. Our present study focused on investigating whether NR2F1-AS1 contributes to the aggressive phenotype of NSCLC cells and showed that the proliferation, migration, and invasion *in vitro* were attenuated and apoptosis induction was promoted in NSCLC cells following NR2F1-AS1 knockdown. Furthermore, the depletion of NR2F1-AS1 suppressed NSCLC tumor growth *in vivo*.

After identifying the expression and functional roles of NR2F1-AS1 in NSCLC, our present study attempted to elucidate the mechanisms underlying the lncRNA-mediated regulation of tumorigenesis in NSCLC. The working theory of lncRNA is that its cellular localization, either in the nucleus or cytoplasm, determines its functional mechanism of action. Therefore, the localization of NR2F1-AS1 in NSCLC cells was determined via subcellular fractionation. NR2F1-AS1 was mostly distributed in the cytoplasm of NSCLC cells. Numerous studies have suggested that lncRNAs can “talk to” miRNAs based on the ceRNA hypothesis [39–41]. LncRNAs can work as ceRNAs and act as a molecular sponge for certain miRNAs, thereby delaying the binding of miRNAs and their target mRNAs, which results in the decrease in the inhibition of target mRNA degradation and/or translation [42].

Our present study used bioinformatics analysis to search for the putative target miRNAs of NR2F1-AS1. A putative binding site of miR-493-5p was identified in the NR2F1-AS1 sequences, which was subsequently validated by luciferase reporter and RIP assays. Moreover, miR-493-5p expression was downregulated in NSCLC tissues and was inversely correlated with NR2F1-AS1 expression. Furthermore, RT–qPCR analysis confirmed that NR2F1-AS1 knockdown increased miR-493-5p expression in NSCLC cells. The following experiments demonstrated that the miR-493-5p-mediated targeting of ITGB1 was positively regulated by NR2F1-AS1 and that the inhibition of miR-493-5p expression can abrogate the regulatory impacts of NR2F1-AS1 knockdown on ITGB1 expression. In summary, these results provided sufficient evidence to identify a ceRNA regulatory axis involving NR2F1-AS1, miR-493-5p, and ITGB1 in NSCLC.

MiR-493-5p was reported to be weakly expressed in NSCLC tissues and positively associated with shorter overall survival in patients with NSCLC [33]. Functional analysis verified the anti-oncogenic activities of miR-493-5p during NSCLC progression. By contrast, ITGB1 expression was upregulated in NSCLC and it functioned as an oncogene [33, 43, 44]. Currently, the molecular mechanisms underlying ITGB1 upregulation and miR-493-5p downregulation in NSCLC cells have not yet been elucidated. The data of our present study revealed high NR2F1-AS1 expression in NSCLC tissues and this expression was negatively correlated with miR-493-5p expression and positively correlated with ITGB1 expression. Furthermore, the interference of NR2F1-AS1 expression resulted in an increase in miR-493-5p expression and a decrease in ITGB1 expression in NSCLC cells. Importantly, rescue assays revealed that the miR-493-5p/ITGB1 axis was the functional mediator of NR2F1-AS1 in NSCLC cells. Consequently, a new regulatory pathway involving NR2F1-AS1, miR-493-5p, and ITGB1 was validated and indicated to perform crucial functions in NSCLC pathogenesis.

## CONCLUSIONS

To the best of our knowledge, our present study highlighted the tumor-promoting roles of NR2F1-AS1 in NSCLC cells for the first time. Mechanistically, NR2F1-AS1 exerted its carcinogenic functions in NSCLC progression by acting as a ceRNA for miR-493-5p and by consequently increasing ITGB1 expression. Our findings may lead to the development of new diagnostic testing and anticancer therapies against NSCLC based on the molecular targets identified.

## MATERIALS AND METHODS

### Patient tissues and cell lines

NSCLC tissues and matched adjacent normal tissues were collected from 73 patients with NSCLC admitted to The Second Xiangya Hospital of Central South University. All samples were obtained from patients who had a single diagnosis of NSCLC and had not been diagnosed with any other forms of cancer at the time of their participation. None of the patients underwent preoperative radiochemotherapy or other antitumor regimens. Patients who received radiotherapy, chemotherapy or other anticancer treatments were excluded from this study. Additionally, patients had been previously diagnosed as other types of human cancer were not admitted in the study. Tissues were quickly immersed in liquid nitrogen after tissue excision and maintained in liquid nitrogen until further analysis.

A normal, nontumorigenic bronchial epithelium cell line—BEAS-2B—was purchased from American Type Culture Collection (ATCC, Manassas, VA, USA) and grown in BEGM^TM^ Bronchial Epithelial Cell Growth Medium (Lonza/Clonetics Corporation, Walkersville, MD). The NSCLC cell lines H522, H460, and H1299 (ATCC) were cultured in RPMI 1640 Media (Gibco; Thermo Fisher Scientific, Inc., Waltham, MA, USA) supplemented with 10% fetal bovine serum (FBS; Gibco; Thermo Fisher Scientific) and 1% penicillin–streptomycin solution (Gibco; Thermo Fisher Scientific). Two other NSCLC cell lines—A549 and SK-MES-1 (ATCC)—were maintained in Ham's F-12K (Kaighn's) Medium and Minimum Essential Medium (Gibco; Thermo Fisher Scientific), respectively, both containing 10% FBS and 1% penicillin–streptomycin solution. All the above mentioned cell lines were maintained at 37°C and placed in a cell culture incubator supplied with 5% CO_2_.

### Transient transfection assay

Three siRNAs that inhibited NR2F1-AS1 expression (si-NR2F1-AS1#1, si-NR2F1-AS1#2 and si-NR2F1-AS1#3) and a negative control siRNA (si-NC) were obtained from Genepharma (Shanghai, China). The MiR-493-5p mimic and miR-493-5p inhibitor (both obtained from Genepharma) were employed to increase and decrease endogenous miR-493-5p expression, respectively. NC miRNA mimic (miR-NC) was considered as the control for the miR-493-5p mimic, and NC inhibitor was considered as the control for miR-493-5p inhibitor. The recombinant pcDNA3.1 integrin β1 (ITGB1) overexpression plasmid (pcDNA3.1-ITGB1; pc-ITGB1) and empty pcDNA3.1 plasmid were obtained from RIBOBIO (Guangzhou, China). The siRNAs (100 pmol), miRNA mimic (100 pmol), miRNA inhibitor (100 pmol) or plasmids (4 μg) were transfected into NSCLC cells using a transfection agent (Lipofectamine 2000, Invitrogen; Thermo Fisher Scientific, Inc.).

### RT–qPCR

Following total RNA isolation using an RNeasy Mini kit (Qiagen GmbH, Hilden, Germany), the purity and concentration of the isolated RNA were determined by measuring the optical density (OD) (A260/A280) using Nanodrop 2000 (Invitrogen; Thermo Fisher Scientific, Inc.). For determining miR-493-5p expression, total RNA was reverse transcribed into complementary DNA using an miScript Reverse Transcription kit (Qiagen GmbH). The synthetic complementary DNA was subjected to qPCR using a miScript SYBR Green PCR kit (Qiagen GmbH). Relative miR-493-5p expression was normalized to U6 small nuclear RNA.

For determining the NR2F1-AS1 and ITGB1 mRNA levels, reverse transcription was performed using a PrimeScript RT Reagent kit (TaKaRa Biotechnology, Dalian, China), and the complementary DNA obtained was used in PCR amplification using a SYBR Premix Ex Taq™ kit (TaKaRa Biotechnology). Glyceraldehyde-3-phosphate dehydrogenase (GAPDH) functioned as the endogenous control for NR2F1-AS1 and ITGB1 mRNA. All data were calculated using the 2^−ΔΔCt^ method. All RT-qPCR primers were shown in Table 2.

**Table 2:** Primer Sequences for RT-qPCR.

**Gene**	**Forward Sequence(5′-3′)**	**Reverse Sequence (5′-3′)**
miR-493-5p	TCGGCAGGUGUACAUGGUAGG	CACTCAACTGGTGTCGTGGA
NR2F1-AS1	AGTACAGGGACTGAGAAACGGAA	TGGTTAATATTGTGGTCACGGAG
ITGB1	TACTTCTGCACGATGTGATGATTTA	ATATCCTCTGGCTTGAGCTTCTCT
U6	CTCGCTTCGGCAGCACA	AACGCTTCACGAATTTGCGT
GAPDH	CGGAGTCAACGGATTTGGTCGTAT	AGCCTTCTCCATGGTGGTGAAGAC

### Subcellular fractionation

A total of 2 × 10^7^ NSCLC cells in their the logarithmic growth phase were collected and extensively rinsed with pre-cooled phosphate-buffered solution, followed by the separation of the cytoplasmic and nuclear fractions using the Cytoplasmic and Nuclear RNA Purification kit (Norgen, Belmont, CA). Subsequent to RNA extraction from both cytoplasmic and nuclear fractions, the distribution of NR2F1-AS1 expression in NSCLC cells was examined via RT–qPCR analysis, as described above.

### CCK-8 assay

Transfected cells were seeded into 96-well plates (2 × 10^3^ cells/well). Cells were maintained at 37°C in a cell culture incubator supplied with 5% CO_2_ for 0, 24, 48, and 72 h. At these time points, 10 μL of CCK-8 reagent (Beyotime, Haimen, China) was added into each well and the cells were further incubated at 37°C for 2 h. OD was determined at 450 nm using an enzyme immunoassay analyzer (Bio-Rad Laboratories, Inc., Hercules, CA, USA).

### Cell apoptosis detection using flow cytometry analysis

The annexin V–fluorescein isothiocyanate (FITC) Apoptosis Detection Kit (Biolegend, San Diego, CA, USA) was used to examine the apoptotic cell population. Trypsinization was performed for harvesting the transfected cells at 48 h posttransfection, following which the cells were washed with ice-cold phosphate-buffered solution and re-suspended in 100 μL staining solution. Thereafter, 5 μL of propidium iodide and 5 μL of annexin V-FITC were added for double-staining. After incubation at room temperature in the dark for 15 min, the apoptotic cell population was identified using flow cytometry (FACScan; BD Biosciences, Franklin Lakes, NJ, USA).

### Cell migration and invasion assays

After culturing for 48 h, FBS-free culture medium was used to prepare transfected cell suspensions. Cell migratory capacity was detected using Transwell chambers with 8-μm pore size membrane inserts (BD Biosciences, Franklin Lakes, NJ, USA). The upper chambers were filled with 200 μL cell suspension containing 5 × 10^4^ cells, whereas 600 μL culture medium containing 10% FBS was added into the lower chambers. At 24 h post-injection, the cells that migrated onto the reverse side of the membranes were fixed using 100% methanol and stained using 0.1% crystal violet; cell that did not migrate and remained on the upper side of membranes were wiped off using a cotton swab. The stained cells were visualized using an inverted microscope (x200 magnification; Olympus Corporation, Tokyo, Japan), and five visual fields were randomly selected for analysis. The experimental procedures of cell invasion assays were the same as those conducted for the cell migration assay, except that the chambers were precoated with Matrigel (BD Biosciences, San Jose, CA). The number of migratory (membrane) and invasive (membrane plus Matrigel) cells was counted and the mean values were used to calculate their migratory and invasive abilities, respectively.

### Xenograft tumor assay

Lentiviruses for small hairpin RNA targeting short hairpin RNA (shRNA) against NR2F1-AS1 (sh-NR2F1-AS1) and scramble negative control shRNA (sh-NC) synthesized by Genepharma were obtained. The lentiviruses were transfected into H460 cells, and the NR2F1-AS1 stably silenced H460 cells were selected via incubation with 1 μg/mL puromycin.

BALB/c male nude mice (4–6-week-old; Model Animal Research Center of Nanjing University; Nanjing, China) were subcutaneously injected with 5 × 10^6^ H460 cells stably expressing sh-NR2F1-AS1 or sh-NC. Each group contained three nude mice. The dimensions of tumor xenografts were monitored every week from day 7 after tumor cell injection. Tumor volume was analyzed using the following formula: tumor volume = 0.5 × length × width^2^. All the mice were sacrificed via cervical dislocation after 5 weeks, and tumor xenografts were excised and weighted. The resected tumor xenografts were subsequently used for RT–qPCR and western blotting.

### Bioinformatics analysis

The target miRNAs of NR2F1-AS1 were predicted using StarBase 3.0.

### RIP assay

The binding of NR2F1-AS1 and miR-493-5p to the AGO2 protein in NSCLC cells was evaluated using the Magna RIP RNA-Binding Protein Immunoprecipitation kit (Millipore, Bedford, MA, USA). NSCLC cells were incubated in a complete RNA immunoprecipitation (RIP) lysis buffer, and the supernatant was treated with RIP buffer containing magnetic beads conjugated with anti-AGO2 or control immunoglobulin G (IgG; Millipore). Following an overnight incubation at 4°C, the magnetic beads were rinsed with a washing buffer, followed by isolation of RNA from the immunoprecipitant complex. The enrichment levels of NR2F1-AS1 and miR-493-5p were detected using RT–qPCR.

### Luciferase reporter assay

The wild-type (wt) NR2F1-AS1 fragment containing the predicted miR-493-5p binding sequences and the mutant (mut) NR2F1-AS1 fragment chemically amplified by Genepharma were obtained and inserted into the psiCHECK-2 luciferase plasmid (Promega, Madison, WI, USA), thus generating the wt-NR2F1-AS1 and mut-NR2F1-AS1 reporter plasmids. These reporter plasmids were transfected into NSCLC cells in parallel with miR-493-5p mimic or miR-NC. At 48 h posttransfection, a Dual Luciferase Reporter Assay System (Promega) was used for the measurement of luciferase activities.

### Western blotting

Cultured cells were collected and lysed in ice-cooled RIPA Lysis and Extraction Buffer (Invitrogen; Thermo Fisher Scientific, Inc.). Bicinchoninic acid assay (Nanjing KeyGen Biotech Co., Ltd; Nanjing, China) was employed to determine the total protein concentration. Sodium dodecyl sulfate–polyacrylamide *gel* electrophoresis (10% gel) was performed for the separation of proteins with equivalent concentrations, following which they were transferred to polyvinylidene fluoride membranes. Blocking was performed by incubating the imprinted membranes for 2 h at room temperature with 5% nonfat dried milk diluted in Tris-buffered saline containing 0.1% of Tween 20. After overnight incubation with primary antibodies at 4°C, a horseradish peroxidase-conjugated secondary antibody (cat. no. ab6721; Abcam, Cambridge, UK) was diluted at a concentration of 1:5000 and further used for incubating the membranes at room temperature for 1 h. The protein bands were developed using ECL Western Blotting Substrate kit (Abcam). The primary antibodies and their sources are as follows: ITGB1 (cat. no. ab52971; Abcam) and GAPDH (cat. no. ab181602; Abcam). GAPDH was used as the loading control.

### Statistical analysis

All experiments were performed in triplicate and repeated at least three times. All results were expressed as mean ± standard deviation. Student’s t-test was used to examine the differences between two groups. Comparisons among ≥3 groups were performed using one-way analysis of variance along with Dunnett’s post-hoc test. Correlations between NR2F1-AS1 and miR-493-5p expressions in 73 NSCLC tissues were tested using Pearson's correlation coefficient. Chi-squared test was used to analyze the association between the NR2F1-AS1 expression and clinical characteristics of 73 patients with NSCLC. The 5-year overall survival of these 73 patients with NSCLC was determined using the Kaplan–Meier method, which was further analyzed with log-rank test. P < 0.05 was considered statistically significant, and P < 0.01 indicated a highly significant difference.

### Ethics Statement

All experimental protocols were approved by the Clinical Research Ethics Committee of The Second Xiangya Hospital of Central South University. Moreover, written informed consent was collected from all participants in the study. Xenograft tumor assay was conducted in accordance with the guidelines of Animal Protection Law of the People’s Republic of China (2009) for experimental animals and with the approval of Ethics Committee of Animal Experiments of The Second Xiangya Hospital of Central South University.
